# SFRP2 is a Novel Diagnostic Biomarker and Suppresses the Proliferation of Pituitary Adenoma

This article has been retracted.

**DOI:** 10.1155/2022/4272525

**Published:** 2022-10-14

**Authors:** Rongxi Huang, Danyan Chen, Hongman Wang, Binghan Zhang, Yu Zhang, Wei Ren

**Affiliations:** ^1^Department of Endocrinology, Chongqing General Hospital, Chongqing, China; ^2^Department of Instrument, Chongqing Emergency Medical Center, Chongqing, China

## Abstract

Pituitary adenoma (PA) constitutes one of the most common intracranial tumors. The present study was designed to identify potential diagnostic markers for PA. We used gene expression profiles (GEO: GSE26966 and GEO: GSE63357 datasets) derived from human PA and nontumor samples that were made freely accessible by the gene expression omnibus (GEO) datasets. Differentially expressed genes (DEGs) were screened between 14 normal specimens and 34 PA specimens by the use of the limma package of the R. The diagnostic genes were determined using a LASSO regression model and SVM-RFE analysis. SFRP2 expression in PA cells was analyzed using RT-PCR, and the effect of SFRP2 dysregulation on PA cell proliferation was measured using CCK-8 analysis. In this study, 361 DEGs were identified: 309 genes were downregulated and 52 genes were upregulated. The results of KEGG assays revealed that the 361 DEGs were mainly enriched in the PI3K-Akt signaling pathway, MAPK signaling pathway, growth hormone synthesis, secretion and action, and AGE-RAGE signaling pathway in diabetic complications. Results from the LASSO regression model and the SVM-RFE analysis indicated that LOC101060391 and SFRP2 were diagnostic genes. In contrast to normal tissue, the expressions of LOC101060391 and SFRP2 were much lower in PA samples. According to the ROC assays, high LOC101060391 and SFRP2 expression had an AUC value >0.9 for PA. Upregulation of SFRP2 distinctly inhibited the proliferative capacity of PA cells, as shown by CCK-8 analysis. Furthermore, knockdown of SFRP2 had an influence on cell growth in both the AtT-20 and HP75 cell lines. Taken together, our findings indicate that LOC101060391 and SFRP2 have diagnostic potential for PA. Furthermore, SFRP2 may be an antioncogene and a therapeutic target for PA.

## 1. Introduction

Pituitary adenoma (PA), accounting for 10%–15% of all cranial tumors, is the third most common brain tumor [1]. Noninvasive pituitary adenocarcinomas (NIPAs), invasive pituitary adenocarcinomas (IPAs), and pituitary adenocarcinomas (PAs) are the three categories that can be used to classify PAs [2, 3]. IPAs have a tendency to infiltrate key surrounding structures, such as the cavernous sinus, the sphenoid bone, and the cranial nerves because of their highly proliferative and invasive nature [4, 5]. When a tumor presses on a nearby organ or tissue, it can create symptoms such as headaches or vision problems, which lead doctors to suspect PAs. This is because PAs do not typically present with the typical symptoms that are associated with hormone hypersecretion [6, 7]. On the other hand, certain tumors have the potential to spread to the cavernous sinus or the region around the internal carotid artery, making it hard to do a total excision [8]. Surgical treatment is beneficial for NFPAs; however, complete removal of certain tumors is not achievable. The purposes of these three different treatment strategies are to lessen or remove the impact of tumor-occupying lesions, rectify excessive hormone release by the tumor, and maintain normal pituitary function [9, 10]. However, after surgery to remove a pituitary tumor, the recurrence rate is rather significant, ranging from 7 to 35 percent [11]. In addition, surgery to remove a pituitary tumor may result in problems such as diabetes insipidus, sphenoid sinusitis, leakage of cerebrospinal fluid, worsening of visual impairment, cerebral palsy, and meningitis [12, 13]. Therefore, it is essential to research and develop effective treatments as well as innovative diagnostic biomarkers.

New disease-related genes have been discovered through the use of microarrays and integrated bioinformatics analysis in recent years. These genes have the potential to operate as biological markers that are diagnostic as well as predictive [14, 15]. For instance, Yang et al. showed that both PVT1 and EZH2 expression levels were elevated in human glioma tissues and cell lines, and this elevation was found to have a positive correlation with the malignancy of the glioma. In addition, inhibiting the expression of PVT1 led to a reduction in cell proliferation, an increase in apoptosis, and a reduction in both migration and invasion via targeting EZH2. In addition, there was a correlation between high expression of PVT1 and a bad prognosis in glioma patients [16]. Huang et al. reported that in patients who had pituitary tumors, the expression of SIRT1 was found to be downregulated in the tumor tissues. The present work indicated, through in vitro tests, that SIRT1 overexpression decreased pituitary tumor cell line growth by inhibiting PTTG1 expression, whereas SIRT1 downregulation demonstrated the reverse effects on pituitary tumor cell line growth [17]. Daniela et al. indicated that the expression of AP52 is significantly increased in gonadotroph and prolactin-secreting pituitary adenomas, where it corresponds with the expression of HMGA2. The above results are in contrast to the expression of AP52 in normal pituitary tissues. RPSAP52 overexpression, from a functional standpoint, stimulated cell multiplication by functioning as a miRNA sponge for HMGA proteins [18]. However, only a few studies have identified the functional genes involved in PA progression. With this study, we aimed to explore the critical diagnostic genes for PA by the use of machine learning.

## 2. Materials and Methods

### 2.1. Cell Culture and Transfection

The HP75 and AtT-20 pituitary tumor cell lines were cultivated in accordance with the instructions provided by the manufacturer. At 37 degrees Celsius and 5% carbon dioxide, the media was supplemented with 1% penicillin-streptomycin and 10% fetal bovine serum (Gibco, USA). AtT-20 and HP75 cells were seeded in six-well plates at the optimal density a full twenty-four hours before the transfection, and the plates were left to incubate overnight. Both AtT-20 and HP75 cells were transfected with pcDNA-SFRP2, sh-SFRP2, and a control (blank plasmid) using Lipofectamine® 3000 reagent and Opti-MEM medium (Invitrogen Life Technologies, USA) in accordance with the methodology provided by the manufacturer. Tolo Biotech was responsible for the procurement of the pcDNA-SFRP2, sh-SFRP2, and blank plasmid (Shanghai, China).

### 2.2. RNA Extraction and Quantitative Real-Time Polymerase Chain Reaction (qRT-PCR)

In order to extract total RNA from cells in accordance with the instructions provided by the manufacturer for qRT-PCR, the FastPure Cell/Tissue Total RNA Isolation Kit V2 was utilized. After completing the reverse transcription of lncRNAs and mRNAs with the help of a reverse transcription system kit, the results were analyzed using quantitative polymerase chain reaction (qPCR) using a Universal SYBR qPCR Master Mix kit. According to the procedure manual, GAPDH was employed in the role of an internal control in order to ascertain the level of mRNAs. For relative quantification, the 2Δ-CT approach was applied. The experiments were repeated three times, and each experiment was triplicated.

### 2.3. Cell Proliferation Assay

After receiving a variety of treatments, the level of cell proliferation was measured utilizing the Cell Counting Kit-8 (CCK-8; TargetMol, Shanghai, China) in accordance with the protocols provided by the manufacturer. To be more specific, 2 × 10^3^ cells were seeded into each well of a 96-well plate, and the plates were then cultured overnight at 37 degrees Celsius and 5% carbon dioxide. Following this, 10 *μ*L of CCK-8 was added to each well. Using a microplate reader set to 450 nm, the optical density of each well was measured. The experiments were repeated three times, and each experiment was triplicated.

### 2.4. Microarray Data

The series of matrix files of the GSE26966 and GSE63357 datasets were obtained from https://www.ncbi.nlm.nih.gov/geo/. The GSE26966 dataset included 9 normal specimens and 14 tumor specimens, whereas the GSE63357 dataset included 5 normal specimens and 20 tumor specimens. The gene symbols corresponding to the probes in each dataset were converted into those symbols using the probe annotation files. When there was more than one probe that corresponded to the same gene symbol, the final expression value of the gene was computed based on the average of all of the probes. Because these two datasets use the same platform and are important for combining data from various datasets, they were combined into a metadata cohort so that additional integration analysis could be performed on the results of the combined datasets. In addition to this, the combat function contained inside the R software's SVA package was utilized in order to eliminate the batch effect.

### 2.5. Data Processing and DEG Screening

After combining the two datasets into a single metadata cohort, the combat function of the SVA package was used to preprocess the data and eliminate any batch effects that may have been present. Differential expression analysis between 14 normal specimens and 34 tumor specimens was all performed with the help of the limma package of the R programming language (https://www.bioconductor.org/). The threshold points for differentially expressed genes (DEGs) were determined to be samples that had an adjusted false discovery rate P that was less than 0.05 and a |log fold change (FC)| that was more than 2.

### 2.6. Gene Functional Enrichment Analyses

Using the “clusterProfiler” R package, functional enrichment was determined in a thorough manner in order to examine the biological activities of DEGs [19]. This was accomplished by detecting gene ontology (GO) word enrichment and KEGG pathway enrichment. The results of the GO enrichment were divided into three categories: molecular functions, biological processes, and cellular components (MF). The GO enrichment and KEGG pathway were determined based on a threshold of *p* value 0.05, and the images that accompany this article represent the top 10 enrichment items.

### 2.7. Candidate Diagnostic Biomarker Screening

Two different machine-learning methods were employed to make predictions about the disease's progression in order to find meaningful prognostic variables. The least absolute shrinkage and selection operator (LASSO) algorithm is a form of regression analysis that makes use of regularization in order to increase the accuracy of prediction [20]. In order to determine the genes that are significantly linked with the differentiation of pituitary tumor samples from normal samples, the LASSO regression technique was implemented in R and run with the “glmnet” package. The support vector machine (SVM) is a popular supervised method of machine learning that may be used for both classification and regression [21]. When selecting the best genes from the metadata cohort, an RFE algorithm was used so as not to fall into the trap of overfitting. Therefore, in order to determine the group of genes that have the greatest capacity for discrimination, support vector machine recursive feature elimination (SVM-RFE) was utilized in order to choose the pertinent characteristics.

### 2.8. Statistical Analysis

The statistical analyses were conducted in the R software (version 3.6.3) and GraphPad Prism 6.0 software. The Student's *t* test and the one-way analysis of variance (ANOVA) were used to compare the data obtained from the various groups. The final data were generated from three independent experiments. *p* values <0.05 were considered statistically significant.

## 3. Results

### 3.1. Identification of DEGs in Pituitary Tumor

In this work, a retrospective analysis was performed on the data obtained from a total of 14 normal specimens and 34 pituitary tumor specimens taken from two different GEO datasets (GSE26966 and GSE63357). After taking into account the batch effects, the DEGs of the metadata were examined with the help of the limma software. 361 DEGs were obtained: 309 genes were downregulated and 52 genes were upregulated (Figures 1(a) and 1(b)).

### 3.2. GO Term and KEGG Pathway Enrichment Analyses of DEGs

To learn more about the biological roles and pathways played by DEGs, researchers can do gene enrichment analysis. As shown in Figure 2(a), the results of GO assays indicated that the 361 DEGs were mainly associated with response to extracellular stimulus, response to nutrient levels, reproductive structure development, response to corticosteroid, endocrine system development, collagen-containing extracellular matrix, endoplasmic reticulum lumen, basement membrane, endosome lumen, photoreceptor outer segment membrane, receptor ligand activity, signaling receptor activator activity, and hormone activity. In addition, the results of KEGG assays revealed that the 361 DEGs were mainly enriched in the PI3K-Akt signaling pathway, MAPK signaling pathway, growth hormone synthesis, secretion and action, and AGE-RAGE signaling pathway in diabetic complications (Figure 2(b)).

### 3.3. Identification of Diagnostic Biomarkers in Pituitary Tumor

In order to search for relevant biomarkers, two different algorithms were utilized. Using the LASSO regression algorithm, the DEGs were narrowed down, and the result was the identification of 15 genes as diagnostic genes for PA (Figure 3(a)). Using the SVM-RFE technique, we were able to choose a subset of three genes from among the DEGs (Figure 3(b)). The two overlapping factors (LOC101060391 and SFRP2) between these two techniques were finally selected (Figure 3(c)). In addition, we analyzed the expressing pattern of LOC101060391 and SFRP2 and found that the expression of LOC101060391 and SFRP2 was noticeably decreased in PA specimens as compared to nontumor specimens (Figures 4(a) and 4(b)). Following that, an investigation into the diagnostic utility of LOC101060391 and SFRP2 in patients suffering from pituitary tumors was carried out. According to the ROC tests, high expression levels of LOC101060391 and SFRP2 exhibited an AUC value that was more than 0.9 for PA (Figures 4(c) and 4(d)).

### 3.4. Effect of SFRP2 on the Growth of Pituitary Tumor Cells in Vitro

The purpose of this study is to investigate the influence that SFRP2 has on the proliferation of HP75 and AtT-20 cells. When compared with the NC group, the findings of the RT-PCR study revealed that the level of expression of SFRP2 was either increased or decreased in HP75 and AtT-20 cells when transplanted with pcDNA-SFRP2 or si-SFRP2, respectively (Figure 5(a)). The findings of the CCK-8 assays revealed that forced SFRP2 expression had a significant inhibiting effect on the ability of AtT-20 and HP75 cells to proliferate in comparison to the NC group (both *p* < 0.05, Figures 5(b) and 5(c)). In addition to this, the effect of SFRP2 knockdown on the proliferation of AtT-20 cells as well as HP75 cells was observed (both *p* < 0.05, Figures 5(b) and 5(c)). As a result of these findings, we hypothesized that an increase in SFRP2 expression could inhibit the growth of pituitary tumors in vitro.

## 4. Discussion

Pituitary tumors come in a variety of subtypes, the most prevalent of which is the prolactin-secreting pituitary adenoma, which accounts for 30–40% of all pituitary tumors [22, 23]. Accompanying this adenoma are headaches, vision problems, irregular periods, enlarged ovaries, infertility, and a lack of sexual desire. Most prolactinomas are benign and respond well to surgical removal, radiation therapy, or drug therapy [24, 25]. Highly effective medications for prolactinoma include cabergoline and dopamine agonists. Pathologically, aggressive prolactin pituitary tumors are intermediate between benign pituitary adenomas and malignant pituitary carcinomas [26, 27]. It is unknown how common malignant prolactin-secreting pituitary tumors are. It is common for them to develop resistance to standard treatments such as TMZ and to experience rapid recurrence after surgery [28, 29]. They have a relatively specific aggressive behavior that is characterized by a marked invasion of surrounding anatomical structures. An extensive study has been carried out in order to investigate the possible biomarkers that could be used for the early diagnosis and treatment of aggressive pituitary tumors. The primary objective of this investigation was to locate previously undiscovered diagnostic biomarkers through the application of machine-learning techniques.

We first evaluated two GEO datasets (GSE26966 and GSE63357) to study the DEGs in PA. After removing the impacts of the batching, the DEGs of the metadata were evaluated by making use of the limma program. Then, we got these results: 309 genes had dramatically decreased expression, while 52 genes had significantly increased expression. To explore the possible function of the 361 DEGs, we performed KEGG assays and found that the 361 DEGs were mainly enriched in the PI3K-Akt signaling pathway, MAPK signaling pathway, growth hormone synthesis, secretion and action, and AGE-RAGE signaling pathway in diabetic complications. Our findings suggest the 361 DEGs may influence tumor progression via regulating the above tumor-related pathways. Importantly, we used two machine-learning methods (LASSO regression algorithm and SVM-RFE) and identified two critical diagnosis genes, including LOC101060391 and SFRP2. Their expression was distinctly decreased in PA specimens compared with nontumor specimens. In addition, ROC assays also confirmed their diagnostic value in screening PA specimens from nontumor specimens. Our findings suggest LOC101060391 and SFRP2 may be used as novel diagnostic biomarkers for PA patients.

SFRP1, SFRP2, SFRP3, SFRP4, and SFRP5 are the five members of the family of proteins known as secreted frizzled-related proteins (SFRP) [30]. It appears that the specific environment plays a role in determining whether the protein known as secreted frizzled-related protein 2 (SFRP2) acts as an antagonist or an agonist for the Wnt signaling pathway [31, 32]. There have been multiple reports of the expression of SFRP2 as well as its function in various cancers. For instance, Wu et al. reported that patients with glioma who were treated with radiotherapy had a decrease in their expression of SFRP2, and this decrease was connected to an advanced stage of the tumor and a bad prognosis. Through the activation of Wnt/-catenin signaling, the CRISP/Cas9-mediated reduction of SFRP2 facilitated the development of soft agar colonies, cancer stemness, and radioresistance in glioma cells [33]. Zhang et al. reported that when compared to the paired adjacent nontumor tissue, the amount of SFRP2 mRNA in NSCLC tissue was found to be significantly lower, while the amount of SFRP2 gene methylation was found to be significantly higher. In addition, the loss of SFRP2 that was mediated by methylation contributed to the increased invasiveness of nonsmall cell lung cancer cells. It was discovered that SFRP2 was weakly expressed in PA, and its knockdown increased the proliferation, migration, and invasion of PA cells by upregulating Wnt signaling [34]. According to these findings, SFRP2 may act as a tumor suppressor in the aforementioned malignancies. In this study, we also found that SFRP2 expression was distinctly decreased in PA specimens, which was consistent with previous findings. However, for the first time, we confirmed SFRP2 as a sensitive diagnostic biomarker for PA based on the results of machine-learning methods. Then, we further performed CCK-8 assays to explore the function of SFRP2 in PA progression and found that its overexpression distinctly suppressed the proliferation of PA cells. It has been known to us that disordered tumor growth is the most important characteristic. Our findings suggest SFRP2 may suppress tumor growth in PA, suggesting it as an antioncogene for PA.

However, our study has a few limitations. First, there were just 14 normal specimens and 34 pituitary tumor specimens combined in the GSE26966 and GSE63357 studies; hence, the sample sizes were quite modest. In a subsequent investigation, there is an urgent need for a larger dataset in order to further validate our results. Secondly, more in vitro and in vivo experiments were needed to further study the function of SFRP2 in the progression of PA.

## 5. Conclusion

We identified two novel diagnostic biomarkers (LOC101060391 and SFRP2) for PA patients. In addition, SFRP2 may be used as a novel therapeutic target for PA.

## Figures and Tables

**Figure 1:** Differentially expressed genes between PA specimens and nontumor specimens. (a) Volcano plot of differentially expressed genes (DEGs). (b) Heat map of the top 100 differentially expressed genes in the analysis result (50 downregulated genes and 50 upregulated genes).

**Figure 2:** Representative results of GO and KEGG analyses. (a) The outcomes of the GO molecular function enrichment, GO cellular component enrichment, and GO biological process enrichment of DEGs. (b) The findings of an examination of DEGs using KEGG pathways.

**Figure 3:** Screening process of diagnostic biomarkers for PA diagnosis. (a) Tuning feature selection in the LASSO. (b) A plot of biomarkers selection via SVM-RFE algorithm. (c) Venn diagram demonstrating two diagnostic markers.

**Figure 4:** The expression of LOC101060391 and SFRP2 in PA and their diagnostic value. ((a) and (b)) The expression of LOC101060391 and SFRP2 was distinctly increased in PA specimens compared with nontumor specimens from GSE26966 and GSE63357 datasets. ((c) and (d)) ROC assays confirmed the diagnostic value of LOC101060391 and SFRP2 for PA based on GSE26966 and GSE63357 datasets.

**Figure 5:** The effect of SFRP2 on the proliferation of AtT-20 and HP75 cells. (a) The RT-PCR method was utilized to analyze the level of SFRP2 expression. ((b) and (c)) The CCK-8 assay was utilized to evaluate the degree to which AtT-20 and HP75 cells were able to proliferate.  ^*∗*^*p* < 0.05 and  ^*∗∗*^*p* < 0.01.

## Data Availability

The original data are provided by the corresponding author upon request without any hesitation.
